# Variations in Soil Microbial Communities and Residues Along an Altitude Gradient on the Northern Slope of Changbai Mountain, China

**DOI:** 10.1371/journal.pone.0066184

**Published:** 2013-06-11

**Authors:** Bin Zhang, Chao Liang, Hongbo He, Xudong Zhang

**Affiliations:** 1 State Key Laboratory of Forest and Soil Ecology, Institute of Applied Ecology, Chinese Academy of Sciences, Shenyang, P. R. China; 2 Graduate University of Chinese Academy of Sciences, Beijing, P. R. China; 3 Department of Soil Science, University of Wisconsin-Madison, Madison, Wisconsin, United States of America; 4 National Field Observation and Research Station of Shenyang Agroecosystems, Shenyang, P. R. China; Wageningen University, The Netherlands

## Abstract

Altitudinally-defined climate conditions provide specific vegetation types and soil environments that could influence soil microbial communities, which in turn may affect microbial residues. However, the knowledge is limited in terms of the degree to which microbial communities and residues present and differ along altitude. In this study, we examined the soil microbial communities and residues along the northern slope of Changbai Mountain, China using phospholipid fatty acid (PLFA) and amino sugar analysis, respectively. Soil samples were taken from five different vegetation belts defined by climates. Principal component analysis (PCA) revealed substantial differences in soil microbial community composition among study sites, appeared to be driven primarily by soil pH and C/N ratio on the first principal component (PC1) which accounted for 50.7% of the total sample variance. The alpine tundra was separated from forest sites on the second principal component (PC2) by a signifiscantly higher amount of fungal PLFA (18:2ω6,9). Soil pH and C/N ratio were also correlated with the ratios of Gram-positive to Gram-negative bacteria (Gm^+^/Gm^−^), glucosamine to galactosamine (GluN/GalN), and glucosamine to muramic acid (GluN/MurA). Both total PLFAs and amino sugars were positively correlated with soil organic carbon, inorganic nitrogen, available phosphorus and potassium. We concluded that soil pH and C/N ratio were the most important drivers for microbial community structure and amino sugar pattern, while substrate availability was of great importance in determining the concentrations of microbial communities and residues. These findings could be used to facilitate interpretation of soil microbial community and amino sugar data derived from measurements in latitude or managed forests.

## Introduction

Soil microorganisms are of great importance to carbon (C) and nitrogen (N) cycling and storage [1], [2], ecosystem functioning [3], and global climate change [4]. Soil microbial communities have consequently received great interests for decades. It is well documented that a number of biotic and abiotic factors, such as vegetation type [5]–[8], temperature [9], water content [10], pH [11], [12], soil type [13], and soil depth [14], influence soil microbial communities, which in turn may affect the turnover and accumulation of soil microbial residues. Our understanding of soil microorganisms and their interactions with environmental factors is improving; however, the influences of climatic regimes on soil microbial communities and residues are still insufficiently investigated, with some existing studies on latitude [15]–[17] but little attention to altitude. The altitudinally-defined vegetation belts on mountain slopes are counterparts to the latitudinally-controlled climatic zones. Temperature gradients in mountains may also represent an analogue to those related to latitude since the mean annual temperature (MAT) decreases with increasing in both altitude and latitude. This makes mountain regions well-suited for the study of climate impacts because of the pronounced climatic gradients on a comparatively small scale [18].

The altitude-induced environmental conditions have been reported to influence soil microbial communities in mountains. For example, a decrease in fungal biomass [19] and diversity [20] with increasing altitude were observed in the Austrian Central Alps. A negative correlation between bacterial population and altitude was reported by Ma et al. [21] in the cold temperate Kalasi Lake and by Giri et al. [22] in a tropical dry deciduous forest. Margesin et al. [19] pointed out several shifts in microbial community composition with altitude in the Austrian Central Alps, such as a significant increase in the relative abundance of fungi and Gram-negative (Gm^−^) bacteria. In contrast, Männistö et al. [23] reported that altitude-varied changes in microbial community composition were controlled by pH rather than temperature fluctuations in Arctic fjelds of Finnish Lapland. Shen et al. [24] also found that soil pH drives the spatial distribution of bacterial communities along elevation on Changbai Mountain with a bar-coded pyrosequencing technique. Moreover, Djukic et al. [25] indicated that the microbial community structure was connected with decomposition conditions and changes in vegetation composition along an elevation gradient in the Austrian Limestone Alps. These studies suggest that soil microbial communities can resist simple prediction and are linked to a wide range of factors than the mere altitude. On the other hand, anabolic activity of microbial communities contributed to soil organic matter (SOM) pool by introducing a mass of the successive refractory residues. The accumulation of microbial residues is highly dependent on the quantity and quality of substrate inputs during laboratory incubation [26]–[28], and several field studies have reported that microbial residues could be preferentially decomposed in soils with poor substrate availability [29], [30]. Different plant species can also specifically influence the contents and patterns of microbial residues in both laboratory and field experiments [29], [31]. Amelung et al. [17] demonstrated a parabolic relationship between the microbial residues and MAT in native grassland soils along a climosequence in North America. Because these factors act in concert along altitude, disentangling their interactions is important for understanding and predicting how soil microbial communities and residues respond to future climate change in mountain soils.

Various methods are available to characterize soil microorganisms. Phospholipid fatty acid (PLFA) analysis is widely accepted as a sensitive tool to indicate viable microbial biomass and fingerprint microbial community composition [32]. Amino sugar analysis is also routinely used to indicate the storage of microbial residues [33]. Furthermore, different origins of individual amino sugars could provide important information on the relative contribution of fungi and bacteria to SOM turnover and accumulation [34]–[36]. The chitin of fungal cell walls is the major source of glucosamine (GluN) in soil, although bacterial cell walls and the exoskeletons of soil invertebrates also make some contribution [37]. Muramic acid (MurA) originates uniquely from bacteria [33], [37]. Despite galactosamine (GalN) accounts for 30–50% of the amino sugar pool, little is known about its origin [28], [36]. Combining viable microbial biomass indicator (PLFAs) and microbial cell wall residues (amino sugars) might provide important information about microbial significance in SOM cycling and storage [38]. However, few studies have considered both methods simultaneously.

The objectives of this study were: (1) to examine soil microbial communities by PLFAs and microbial residues by amino sugars along an altitude gradient of Changbai Mountain; (2) to determine if and how differences in soil microbial communities and residues are correlated with environmental factors; and (3) to explore the control and feedback between PLFAs and amino sugars.

## Materials and Methods

### Study area and soil sampling

This study was conducted on the northern slope of Changbai Mountain in Jilin Province, northeastern China (Figure 1). The permission is issued by Changbai Mountain Administrative Committee. According to the Köppen Climate Classification, the climate of this region is humid continental. From the lowest part of the mountain at 740 m to the summit at 2691 m, the MAT decreases from 2.8 to –7.3°C, the mean annual precipitation (MAP) increases from 750 to 1340 mm [39]. Climatic and topographic variations along the altitude gradient result in five vertical vegetation belts on the northern slope (Figure 1). Therefore, five study sites (one in each vegetation belt) were selected to represent a climosequence from the montane ecosystems to the subalpine and alpine zones (Figure 1, Table 1). The influence of human activities was minimized by selecting sites that have not been disrupted.

**Figure 1:** Map of study area and the five vertical vegetation belts along the northern slope of Changbai Mountain, China. The locations of the study sites were marked with rectangles.

**Table 1:** Site information and general soil characteristics.

Site	Altitude (m)	Coordinates	Vegetation	MAT^a^ (°C)	MAP^a^ (mm)	SOC^a^ (mg g^−1^)	C/N	pH (H_2_O)	NH_4_+NO_3_ (mg kg^−1^)	P (mg kg^−1^)	K (mg kg^−1^)
1	807	42°23′ N 128°05′ E	Broadleaved and Korean pine forest	2.58	691	171a^b^	14.9c	5.10a	123a	27.2a	300a
2	1204	42°09′ N 128°09′ E	Korean pine and spruce-fir mixed forest	0.27	811	59.6d	19.4b	4.57c	53.0c	13.2c	173c
3	1707	42°04′ N 128°04′ E	Dark coniferous forest	−2.29	967	96.5b	21.2a	3.95d	55.8c	11.3d	173c
4	1974	42°03′ N 128°04′ E	Erman’s Birch forest	−3.31	1038	65.4c	15.4c	4.59c	79.3b	8.10e	163d
5	2295	42°02′ N 128°04′ E	Alpine tundra	−4.84	1154	59.5d	18.6b	4.78b	57.9c	16.2b	180b

a MAT, mean annual air temperature; MAP, mean annual precipitation; SOC, soil organic carbon.

b Different letters within each column indicate significant differences among study sites (*P*<0.05, Tukey’s HSD)

Four replicate soil monoliths (25×25 cm) were collected from each of the five sites on July 20, 2009. Samples were taken from the A horizon after the litter and humus layer was removed carefully. The horizon thickness varied from 5 to 11 cm. Field-moist samples were placed in a plastic bag and kept cool until processed in the laboratory. After removal of visible fresh roots and plant material, the soils were homogenized and passed through a 2-mm sieve. One sub-sample was air-dried for soil chemical analyses. Another sub-sample was freeze-dried and used for PLFA extraction.

### Soil chemical analyses

Soil total C and N were determined by dry combustion on ground samples (100-mesh) using a C/N analyzer (LECO Corporation, MI, USA). Because these soils are free of carbonates, the total C content is equivalent to soil organic C (SOC) content. Soil pH was measured in a 1:2.5 soil/water suspension. Available phosphorus (P) and potassium (K) were determined, respectively, by Bray-1 method and ammonium acetate extraction method [40]. NH_4_ and NO_3_ were extracted with 2 M KCl and analyzed on a TRAACS 2000 autoanalyzer by using the Berthelot reaction method and cadmium reduction method, respectively.

Amino sugar analysis was conducted according to Zhang and Amelung [41]. Briefly, samples were hydrolyzed with 6 M HCl at 105 °C for 8 h, and then the solution was filtered and purified by neutralization. After drying of the supernatant, amino sugars were washed out from the residues using methanol, transformed into aldononitrile derivatives, and then extracted from the aqueous solution with dichloromethane. The amino sugar derivatives were separated on an Agilent 6890A gas chromatography (GC, Agilent Technologies, USA) equipped with an HP-5 capillary column (30 m×0.32 mm×0.25 µm) and a flame ionization detector (FID). Amino sugars were quantified based on the internal standard myo-inositol which was added prior to purification. Methyl-glucamine was used as a recovery standard before derivatization to monitor recovery efficiency. We calculated the total amino sugar content as the sum of the four amino sugars determined. We used GluN as the biomarker for fungal cell-wall residues and MurA for bacterial cell-wall residues. Mannosamine (ManN) is not considered alone due to its ambiguous origin and trace amounts.

### Phospholipid fatty acid analysis

PLFA extraction was conducted for each sample following the procedure of Bligh and Dyer [42] after modifications by Bossio et al. [13]. Briefly, lipids were extracted in a single-phase chloroform-methanol-citrate buffer (1∶2∶0.8) system. Phospholipids were separated from neutral lipids and glycolipids on silica solid phase extraction columns (Supelco, Inc., Bellefonte, USA). After methylation of the polar lipids, PLFA methyl esters were analyzed by an Agilent 6890A GC equipped with an HP-5 capillary column (30 m×0.32 mm×0.25 µm) and a FID. Nonadecanoic acid methyl ester (19∶0, Sigma-Aldrich) was added as an internal standard when the samples were dissolved in 150 µL of hexane before GC analysis. Super purified nitrogen was used as the carrier gas with a flow rate of 0.8 mL min^−1^. The Supelco 37 Component FAME Mix and Bacterial Acid Methyl Esters (Sigma-Aldrich) were used for peak identification and quantification. A total of thirty-four different PLFAs including saturated, monounsaturated, polyunsaturated, cyclopropyl, and methyl fatty acids were identified. Fifteen PLFAs (14:0, i15:0, a15:0, 15:0, i16:0, 16:1ω7c, 16:0, i17:0, cy17:0, 17:0, 18:2ω6,9, 18:1ω9c, 18:1ω9t, 18:0, 20:0) consistently presented in the samples were used for data analysis. The fatty acid signatures 14:0, i15:0, a15:0, 15:0, i16:0, 16:1ω7c, i17:0, cy17:0, and 17:0, which are considered to be of bacterial origin [32], were used as biomarkers for bacterial biomass. The fatty acid 18:2ω6,9, which is known to correlate well with ergosterol, was used as an indicator for fungal biomass [32]. We used fatty acids i15:0, a15:0, i16:0, and i17:0 to represent Gram-positive (Gm^+^) bacteria, whereas cy17:0, 16:1ω7c, 14:0, 15:0, and 17:0 to represent Gm^−^ bacteria [25]. The sum of all PLFAs was used to represent total microbial lipid biomass.

### Statistical analyses

To explore variation in soil microbial community composition among study sites, the mole percentages (mol%) of individual PLFAs were subjected to principal component analysis (PCA) after standardizing to unit variance. To explore the relationships between individual PCs and environmental variables, redundancy analysis (RDA) was carried out with the rda function in the ‘vegan’ library in R. One-way analysis of variance (ANOVA) procedures, with Tukey’s honestly significant difference (HSD) as post hoc, were used to test significant differences in soil properties, sums and ratios of various microbial lipid groups, and concentrations and patterns of amino sugars among study sites. Correlations between variables were calculated with the Pearson correlation coefficients. Statistical analysis was performed using the software package SPSS 13.0 for Windows (SPSS Inc. Chicago, USA). Figures were generated by Sigmaplot 10.0 (Systat Software Inc.) and the R package.

To explore the amino sugar data explained by a linear model of individual PLFAs and soil properties, RDA was carried out again. The ordination of the response variables (amino sugar data) was constrained by a multiple regression on the explanatory variables (individual PLFAs and soil properties).The explanatory PLFAs were selected by three rules: (1) significantly correlated with individual amino sugars; (2) indicative of specific microbial groups; and (3) higher in mol% (>5%). NO_3_, K, and P were excluded from the explanatory variables as they were significantly correlated with SOC. The significance of the RDA results was tested by permutation test (999 permutations). Since *P*<0.001, we presented the ordination biplot which shows sites as points, amino sugars, individual PLFAs, and soil properties as vectors. The angles in the biplot between response and explanatory variables, and between response variables themselves or explanatory variables themselves, reflect their correlations. The proportion of explained variation was calculated by using adjusted R-squared values as described by Peres-Neto et al. [43]. The biplot was generated by the R package.

## Results

### Soil characteristics

Selected soil characteristics were significantly different among study sites (*P*<0.05, Table 1). Although MAT decreases and MAP increases with increasing elevation, there was no altitudinal changing trend for these soil properties. However, if we excluded site 2 from the study sites, a significant decrease was observed in SOC with increasing altitude (*P*<0.05, Table 1). The C/N ratios varied from 14.9 to 21.2, with the lowest value found at the site that is dominated by broadleaf trees (site 1) and the highest at the site with the highest percentage of conifers (site 3). All study sites were acidic (Table 1). The lowest soil pH (3.95) was found at the site with the highest C/N ratio (site 3) and the highest (5.10) at the site with the lowest C/N ratio (site 1). Soil available P, K, and inorganic N (NH_4_ + NO_3_) ranged from 8.10–27.2, 163–300, and 53.0–123 mg kg^−1^, respectively (Table 1).

### Phospholipid fatty acids

Total microbial lipid biomass was significantly higher in site 1 (302 nmol g^−1^ soil) and significantly lower in sites 2, 4, and 5 (125–129 nmol g^−1^ soil) in comparison with site 3 (195 nmol g^−1^ soil, *P*<0.05). Total microbial lipid biomass was positively correlated with SOC (*r* = 0.99, *P*<0.01), inorganic N (*r* = 0.80, *P*<0.01), available P (*r* = 0.81, *P*<0.01) and K (*r* = 0.92, *P*<0.01).

Principal component analysis of the PLFA data suggested substantial differences in soil microbial community composition among study sites (Figure 2A). The first principal component (PC1) explained 50.7% and the second (PC2) 26.4% of the total variance in the PLFAs. PC1 was negatively correlated with soil pH (*r* = –0.92, *P*<0.001) and positively with C/N ratio (*r* = 0.82, *P*<0.001) (Figure 2C). The site with the highest pH and lowest C/N ratio (site 1) was found on the left-hand side of Figure 2A, the sites with intermediate pH values and C/N ratios (sites 2, 4, and 5) in the middle portion of Figure 2A, and the site with the lowest pH and highest C/N ratio (site 3) on the right-hand side of Figure 2A. Along the PC2 axis, the alpine tundra (site 5) showed negative scores, while the forest sites (sites 1–4) showed positive scores. The PCA plot also showed that data points for sites 2 and 4 were intermixed (Figure 2A). For PC1, lipid signatures i15:0, 16:0, and 16:1ω7c had higher positive loading scores while a15:0 had lower negative loading scores (Figure 2B). For PC2, the fungal biomarker 18:2ω6,9 had large negative loading scores and appeared to become less abundant in sites 1–4 than site 5 (Figure 2B).

**Figure 2:** Multivariate statistical analysis of the phospholipids fatty acids (PLFAs) data. A) Principal component analysis (PCA) of PLFAs (mol%) in different study sites along an altitude gradient on the northern slope of Changbai Mountain, China. PC1 explains 50.7% of the variance in the PLFA data, PC2 explains 26.4%. Sites 1–5 represent a climosequence from the montane to the subalpine and alpine vegetation zones. B) Loading plot for individual PLFAs. The PLFAs most responsible for the variations in soil microbial community composition among study sites were presented by vectors. C) Redundancy analysis (RDA) ordination biplot showing relationships between the first two PCs and environmental variables. The environmental variables followed by an asterisk indicate significant influences on the PCs. Environmental variables are scaled by the blue dashed axes. SOC, soil organic carbon; TN, total nitrogen; MAT, mean annual air temperature; MAP, mean annual precipitation.

The absolute abundance of specific microbial groups showed different patterns along the altitude gradient. Site 1 contained 31.9% higher (*P*<0.05) bacterial PLFAs than site 3, while it had similar concentration of fungal PLFA as site 3 (Figure 3). Both bacterial and fungal PLFAs in sites 2 and 4 were similar (*P*>0.05), but significantly lower than those in sites 1 and 3 (*P*<0.05, Figure 3). Site 5 had the highest fungal PLFA and lowest bacterial PLFAs, which resulted directly in significantly higher fungi to bacteria (F/B) ratio than other sites (*P*<0.05, Figure 3). Significantly higher F/B ratios were also observed in sites 2 and 3 than sites 1 and 4 (*P*<0.05, Figure 3). The ratios of Gm^+^/Gm^−^ were significantly lower in sites 3 and 5 than sites 1, 2, and 4 (*P*<0.05, Figure 3).

**Figure 3:** Sums and ratios of phospholipid fatty acids (PLFAs) of various microbial groups in different study sites along an altitude gradient on the northern slope of Changbai Mountain, China. Different letters within each group indicate significant differences among study sites (*P*<0.05, Tukey’s HSD). Error bars show standard errors (n = 4). F/B, the ratio of fungal to bacterial PLFAs; Gm^+^/Gm^−^, the ratio of Gram-positive to Gram-negative bacteria.

### Amino sugars

For the study sites, the concentrations of individual amino sugars varied from 1793 to 7205 µg GluN g^−1^ soil, from 586 to 2431 µg GalN g^−1^ soil, and from 105 to 413 µg MurA g^−1^ soil (Figure 4). All three amino sugars had significantly greater concentrations at site 1 (*P*<0.05). GluN was significantly higher in sites 3 and 4 and significantly lower in site 5 compared with site 2 (*P*<0.05), while GalN decreased in the order site 4> site 3> site 5> site 2 (Figure 4). MurA was not significantly different among sites 2–5 (*P*>0.05, Figure 4). Both GluN/GalN and GluN/MurA ratios were significantly higher in sites 2 and 3 than sites 1 and 5 (*P*<0.05, Figure 4). Site 4 had similar GluN/GalN ratio as sites 1 and 5 and similar GluN/MurA ratio as sites 2 and 3 (*P*>0.05, Figure 4). Total amino sugars varied in the same way as GluN did, with values ranging from 2656 to 10357 µg g^−1^ soil, and were positively correlated with SOC (*r* = 0.97, *P*<0.01), inorganic N (*r* = 0.91, *P*<0.01), available P (*r* = 0.84, *P*<0.01), and available K (*r* = 0.97, *P*<0.01). Total amino sugar amounts in SOC (AS/SOC) were significantly higher in sites 1 and 4 (60.5 and 59.5 mg g^−1^ respectively) and significantly lower in sites 3 and 5 (40.1 and 44.7 mg g^−1^ respectively) in comparison with site 2 (54.0 mg g^−1^, *P*<0.05).

**Figure 4:** Concentrations and patterns of amino sugars in different study sites along an altitude gradient on the northern slope of Changbai Mountain, China. Different letters within each group indicate significant differences among study sites (*P*<0.05, Tukey’s HSD). Error bars show standard errors (n = 4). GluN, glucosamine; GalN, galactosamine; MurA, muramic acid.

### Relationships between amino sugars and PLFAs

RDA showed that the first and second canonical axes explained 28.6% and 7.3%, respectively, of the total variance in the amino sugar data (Figure 5). Because ecological data are generally quite noisy, we can be confident that the major trends have been modeled in this analysis. Furthermore, the first unconstrained eigenvalue is comparatively small, which means that it does not display any important residual structure of the amino sugar data. The amino sugar data appeared to fall into two groups in the ordination biplot, which can be described as: (1) fungal-derived GluN; and (2) GalN and bacterial-derived MurA. Both groups seemed positively correlated with a15:0, i17:0, SOC, and TN. Permutation test by terms revealed a15:0, i15:0, i16:0, i17:0, 16:1ω7c and SOC had significant influence on amino sugar data. In addition, the study sites in the ordination biplot were clearly separated.

**Figure 5:** Redundancy analysis (RDA) of the amino sugar data for 20 soil samples using 7 microbial lipids and 7 environmental properties as explanatory variables. The amino sugars and sites are scaled by the black solid axes (bottom and left), and the explanatory variables are scaled by the blue dashed axes (top and right). The explanatory variables followed by an asterisk indicate significant influences on the amino sugar data.The proportion of explained variation was calculated by using adjusted R-squared values as described by Peres-Neto et al. [43]. GluN, glucosamine; GalN, galactosamine; MurA, muramic acid; SOC, soil organic carbon; TN, total nitrogen; MAT, mean annual air temperature; MAP, mean annual precipitation.

## Discussion

In this study, we examined soil microbial communities and residues along an elevation gradient of Changbai Mountain. We found neither soil microbial communities nor residues showed a consistent altitudinal change along the studied elevation gradient. Similar altitudinal trends in microbial communities were found in Austrian Limestone Alps [25] and Bornean tropical forest ecosystems [44]. In contrast, Margesin et al. [19] observed a decrease of microbial (bacterial and fungal) biomass with increasing altitude in the Austrian Central Alps. One possible explanation for the apparent disparity between studies lies in site selection. For example, Djukic et al. [25] selected six study sites in 200-m elevation increments from 900 to 1900 m, whereas Margesin et al. [19] compared microbial communities only between alpine (2300–2530 m) and subalpine (1500–1900 m) soils. Because there was no available study regarding microbial residues along altitude, we compared our amino sugar data with the results from latitudinal studies. While Sowden [45] did not find any correlation between amino sugars and climatic elements in Canadian soils from different climate and vegetation zones, Amelung et al. [17] showed a parabolic relationship between amino sugars and MAT along a climosequence in North America. It seems that the effect of altitude on soil microbial communities and residues was indirect and mainly through its control on vegetation inputs and microbial habitat in our study. Alternatively, it could be that the control mechanism of altitude was more complex than simple linear relationship.

This study indicated that soil pH and C/N ratio were the most important drivers for soil microbial community composition and residue pattern along the northern slope of Changbai Mountain. Similar forces were found to shape microbial community composition in boreal forest soils [46] and alpine environments [25]. This is also in agreement with the results observed by ribosomal RNA gene based analysis on the same mountain [24]. The site with the lowest pH and highest C/N ratio (site 3) was structurally distinct from the other sites as a consequence of higher relative abundance of i15:0, 16:1ω7c, and 16:0 and lower relative abundance of a15:0. Significantly higher i15:0/a15:0 ratio (3.75) in this site than other sites (1.57–1.71) indicated niche stress for microbial growth. This is in line with report of increased i15:0 and decreased a15:0 in low pH oak forest soils [47]. However, Nilsson et al. [47] also found the PLFA 16:1ω7c was associated with high pH in forest soils, which seems to contrast with our results. Disparities might be explained if other methods determining microbial community composition at higher resolution were included, such as ribosomal RNA gene based analysis [24]. The lower Gm^+^/Gm^−^ ratio in this site probably contributed to its higher GluN/MurA ratio because cell wall of Gm^−^ bacteria contains thinner murein layers than that of Gm^+^ bacteria, leading to lower MurA concentrations in living Gm^−^ than Gm^+^ bacteria [48], [49].

It is generally held that soils with high pH and low C/N ratio are more favourable to bacteria than fungi, and vice versa [50], [51]. This supports our result of fungal dominance at sites 2 and 3 and bacterial dominance at sites 1 and 4 (Figure 3, Table 1). Our observations are consistent with reports of increased F/B ratios in low pH coniferous forest soils than in high pH beech forest soils [32]. The influence of soil pH and C/N ratio on the relative abundance of fungi and bacteria in the studied forest sites was well reflected in GluN/GalN ratio (Figure 3, 4). An increasing GluN/GalN ratio has been used to indicate an increasing fungal contribution to SOM humification in forests [37]. Liang et al. [38] reported that of three forest soils, the one with the highest F/B ratio showed the highest fungal contribution to the soil amino sugar pool, which is in line with our study. However, such reflection was not observed in heavy metal polluted soils [52] or agricultural soils under contrast tillage practices [53]. Our results substantiate the “memory effect” of microbial residues which integrate microbial community structure over time [28], [54].

A negative correlation was found between C/N ratios and the ratios of total amino sugars to total PLFAs (*r* = −0.86, *P*<0.01). This corresponds well with the study of Liang et al. [38] in which a decrease in the ratio of amino sugars to PLFAs was associated with an increase in C/N ratio. This result could be explained by selective preservation which is a common humification pathway in forest soils [55]. For example, site 3 contained a relatively higher living biomass (Figure 3). However, due to the poor quality of substrate (C/N ratio, 21.2), amino sugars might be decomposed and served as a preferred substrate for microorganisms to meet their growth needs. This is also the case for sites 2 and 5 with C/N ratios of 19.4 and 18.6, respectively, resulting in significantly lower microbial contribution to SOM pools (AS/SOC) in those sites than sites 1 and 4.

The significant correlation between nutrient availability and PLFAs as well as amino sugars indicated a strong substrate control over microbial communities and their residues. Substrate availability was also found to influence soil microbial communities in Bornean tropical forests [44] and soil microbial residues in a Michigan old-growth forest [29]. Soil microorganisms are usually considered to be C limited [56], even in coniferous forest soils with high soil C/N ratios [57] such as site 3 of our study. In this study, individual amino sugars contributed to the total in the order GluN > GalN > MurA, which is consistent with results from other forest soils [29], [58], native grassland soils [17], and agricultural soils [30], [59].

Despite a few studies found significant tree species-specific effects on soil microbial communities [5], [6] and residues [29], we put less focus on vegetation since Ushio et al. [60] pointed out tree species influence soil microbial community mainly through their effects on soil pH, total C and N. Nevertheless, the fungal dominance of the coniferous forests (sites 2 and 3) in our study could be partially explained by vegetation types. Fungi are thought to be more efficient in the decomposition of recalcitrant phenolic compounds [6] which have been identified with high quantities in coniferous forest [61]. In addition, ectomycorrhizal fungi could partially contribute to the fungal biomass since they exist in a symbiotic relationship with various species of coniferous trees [62].

The findings of this research also provide some insight into the relationships between soil microbial communities and their residues, as indicated by the relationships between the PLFA and amino sugar signatures in the ordination biplot. The positive correlations of amino sugars with bacterial-derived PLFAs suggest that variations in bacterial communities could lead to changes in amino sugars. It seems that bacteria, especially Gm^+^ bacteria, played a more important role in the turnover and accumulation of amino sugars. The significant correlation between Gm^+^/Gm^−^ and AS/SOC (*r* = 0.83, *P*<0.01) supports this point. Fungal PLFA 18:2ω6,9, on the other hand, did not show a significant influence on amino sugar data despite the fungal-derived GluN accounted 67.5–76.5% of the total amino sugar pool. The significant influence of SOC on amino sugar data is consistent with the substrate control discussed above. Nevertheless, it remains a significant challenge to determine how the changes in microbial communities that occur under different environmental conditions could be manifested in changes in microbial residues.

## Conclusions

In this study, we examined soil microbial communities and residues along an elevation gradient of Changbai Mountain by analyzing PLFA and amino sugar signatures. We found both soil microbial communities and residues differ between sites, thus reflecting variations between sites in several biotic and abiotic factors. However, the differences were not related to altitude, suggesting either the control of altitude is indirect or the mechanism is complex than simple linear relationship with soil microbial communities and residues. We found soil pH and C/N ratio were the most important drivers for microbial community structure and amino sugar pattern, while substrate availability was of great importance in determining the concentrations of microbial communities and residues. Redundancy analysis indicated bacteria were more important in controlling the feedback with amino sugar pools than fungi.
